RETRACTED

# Clinical Value of PLR, MLR, and NWR in Neoadjuvant Chemotherapy for Locally Advanced Gastric Cancer

**DOI:** 10.1155/2022/8005975

**Published:** 2022-05-26

**Authors:** Baojun He, Jieli Wu

**Affiliations:** ^1^Department of Clinical Laboratory Medicine, The First Affiliated Hospital of Jinzhou Medical University, Jinzhou, Liaoning 121001, China; ^2^Department of Oncology Medicine, The First Affiliated Hospital of Jinzhou Medical University, Jinzhou, Liaoning 121001, China

## Abstract

**Objective:**

The clinical value of platelet-to-lymphocyte ratio (PLR), monocyte-to-lymphocyte ratio (MLR), and neutrophil-to-white blood cell ratio (NWR) in predicting the prognosis of patients with locally advanced gastric cancer after neoadjuvant chemotherapy (NACT) was studied.

**Methods:**

A total of 131 patients with locally advanced gastric cancer treated with neoadjuvant chemotherapy in our hospital from May 2015 to June 2018 were selected as the study subjects, and all were treated with neoadjuvant chemotherapy. The relationship between the values of PLR, MLR, and NWR and the efficacy of neoadjuvant chemotherapy and clinical staging was analyzed; all patients were followed up for 3 years. Patients were divided into death group and survival group according to the survival of patients. The predictive value of PLR, MLR, and NWR values for patients' prognosis was analyzed, and the survival rates of patients with different PLR, MLR, and NWR values were compared.

**Results:**

The effective rate of neoadjuvant chemotherapy in patients with locally advanced gastric cancer was 62.60% (82/131), and the PLR, MLR, and NWR values in the effective group were lower than those in the ineffective group (*P* < 0.05). The AUC of combined PLR, MLR, and NWR in evaluating the efficacy of neoadjuvant chemotherapy was greater than that of PLR and NWR alone (*P* < 0.05). The PLR value of patients with stage IIIa, IIIb, and IIIc was greater than that of patients with stage II, the MLR value of patients with stage IIIb and IIIc was greater than that of patients with stage II and IIIa, and the NMR value of patients with stage IIIc was greater than that of patients with stage II, IIIa, and IIIb (*P* < 0.05). PLR, MLR, and NWR values were positively correlated with clinical stage (*P* < 0.05). The PLR, MLR, and NWR values in the survival group were lower than those in the death group (*P* < 0.05). The AUC of combined PLR, MLR, and NWR in predicting the prognosis of patients was greater than that of MLR and NWR alone (*P* < 0.05). The survival rate of patients with PLR ≥ 162.11 (36.21%) was lower than that of patients with PLR < 162.11 (80.82%), and the survival rate of patients with MLR ≥ 0.31 (42.86%) was lower than that of patients with MLR < 0.31 (74.67%), and the survival rate of patients with NWR ≥ 0.62 (45.00%) was lower than that of patients with NWR < 0.62 (74.65%) (*P* < 0.05).

RETRACTED

**Conclusions:**

PLR, MLR, and NWR values are correlated with clinical stage, and the combined detection has value in evaluating the clinical efficacy of neoadjuvant chemotherapy and predicting the prognosis of patients with locally advanced gastric cancer.

## 1. Introduction

Gastric cancer is a common malignant tumor of the digestive system, with a high incidence in East Asia. Surgery is the most effective method for the treatment of gastric cancer. The 5-year survival rate after radical resection of early gastric cancer can reach over 90%, but early gastric cancer usually has no obvious symptoms, which cannot cause patients to pay attention to it. When patients can feel obvious symptoms, the lesions are already in advanced stage [1]. Neoadjuvant chemotherapy (NACT) has become an important means for the treatment of intermediate and advanced cancer. The use of NACT in the treatment of locally advanced gastric cancer can effectively play a role in tumor downstaging, improve the rate of radical surgery for patients with advanced gastric cancer, improve the quality of life of patients, and improve the prognosis of patients [2, 3]. According to the diagnosis and treatment guidelines of the Collaborative Professional Committee of Clinical Oncology of the Chinese Anti-Cancer Society, clinical diagnosis and prognosis assessment of gastric cancer patients mainly rely on imaging, pathological, gastroscopy, and immunohistochemical examinations [4]. However, whether there are more convenient indicators to evaluate the prognosis of patients deserves further discussion. Inflammatory response is closely related to the occurrence and development of tumors. Inflammatory cells can regulate the tumor microenvironment by releasing a variety of cytokines, promote the proliferation of tumor cells, inhibit their apoptosis, promote the distant metastasis of tumor, and affect the prognosis of tumor patients [5]. According to relevant studies, the white blood cells, platelets, lymphocytes, peripheral blood neutrophils, platelet-to-lymphocyte ratio (PLR), and neutrophil-to-white blood cell ratio (NWR) are closely related to tumor prognosis, PLR can reflect the level of systemic inflammation in patients and can be used to evaluate the prognosis of gastric cancer patients [6]. Since the lymph node stage (pN) of UICC clinical tumor stage (TNM) may have obvious “stage deviation” phenomenon, which can directly affect the prognosis evaluation of gastric cancer, some studies have used the monocyte-to-lymphocyte ratio (MLR) to predict the prognosis of gastric cancer patients, which has certain predictive value [7]. The purpose of this study was to investigate the clinical value of PLR, MLR, and NWR in predicting the prognosis of patients with locally advanced gastric cancer treated with neoadjuvant chemotherapy, which is reported as follows.

RETRACTED

## 2. Materials and Methods

### 2.1. General Information

A total of 131 patients with locally advanced gastric cancer who received neoadjuvant chemotherapy in the hospital from May 2015 to June 2018 were selected as the study subjects, including 79 males and 52 females. The age ranged from 41 to 65 years, with an average of 52.17 ± 6.09 years. This study was approved by the hospital ethics committee.

### 2.2. Inclusion Criteria

(1) All patients were diagnosed as gastric cancer by postoperative pathological diagnosis [8, 9]. (2) All patients could tolerate surgical resection and drug chemotherapy. (3) There were measurable lesions.

### 2.3. Exclusion Criteria

The exclusion criteria are as follows: (1) patients with serious complications during hospitalization; (2) patients who had received chemotherapy before enrollment; (3) patients with incomplete clinicopathological data; (4) patients with serious infections or immune system diseases; (5) patients combined with other malignant tumors; (6) patients combined with severe organ dysfunction such as the heart, liver, and kidney; and (7) patients with estimated survival time of < 3 months

### 2.4. Methods

#### 2.4.1. Treatment Methods

All patients were given neoadjuvant chemotherapy. The chemotherapy regimen was MFOLFOX6, oxaliplatin 85 mg/m^2^ was given intravenously for 2 hours on the first day, fluorouracil 0.4 g/m was given continuously intravenously (after calcium tetrahydrofolate), and fluorouracil 2.4 g/m^2^ was given continuously intravenously for 46 hours (perfusion by chemotherapy pump). It was repeated every 2 weeks, and the lesions were evaluated by CT after 2-3 cycles. For patients with reduced lesions, surgery was performed after 2 weeks of rest. For patients with intraoperative ascites, the ascites was extracted for centrifugation, and exfoliated cytology was performed. For those without ascites, the abdominal cavity was rinsed with normal saline and then centrifuged with washing fluid. If no cancer cells were found, surgical resection was performed. The resection range included the whole stomach and left lobe of the liver, with the resection margin referring to the principle of radical tumor resection of the organ where the tumor was located. Infection prevention and nutritional support were performed in the perioperative period, and postoperative treatment was performed by an oncologist based on the original protocol for a total of 12 cycles. For those who respond to chemotherapy, symptomatic treatment was performed.

RETRACTED

#### 2.4.2. Clinical Efficacy Evaluation

According to the “Response Evaluation Criteria in Solid Tumors (RECIST)” [10], patients were divided into complete remission, partial remission, stable disease, and disease progression. Partial remission means that the reduction of the tumor by more than 50% (in the case of a single tumor, the product of the longest diameter of the tumor and its largest vertical diameter is reduced by more than 50%; in the case of multiple tumors, the sum of the areas of multiple tumors is reduced by more than 50%). Stable disease means that the tumor area decreases by less than 50% or increases by less than 25%. Partial remission means that the tumor increases by more than 25% or new lesions appear. Complete remission and partial remission were defined as effective. According to this, the enrolled patients were divided into effective group and ineffective group.

#### 2.4.3. Prognosis Evaluation

The survival of patients was followed up for 3 months, 6 months, 1 year, 2 years, and 3 years by telephone or outpatient follow-up. Patients were divided into death group and survival group according to 3-year survival after treatment.

#### 2.4.4. Detection of PLR, MLR, and NWR Values

Fasting venous blood was collected from patients before treatment; platelet, lymphocyte, neutrophil, white blood cell, and monocyte counts were detected by Sysmex XE-2100 hematology analyzer (Sysmex Corporation, Japan); and PLR, MLR, and NWR values were calculated.

### 2.5. Observation Indicators

(1) The PLR, MLR, and NWR levels of the effective group and the ineffective group were compared, and the evaluation value of PLR, MLR, and NWR levels on clinical efficacy was analyzed. (2) The patients were staged according to the TNM staging system for gastric cancer promulgated by the International Union Against Cancer (UICC) and the American Joint Oncology (AJCC). PLR, MLR, and NWR levels of patients with different clinical stages were compared to analyze the correlation between PLR, MLR, and NWR levels and clinical stage. (3) PLR, MLR, and NWR levels were compared between the survival group and the death group, and the predictive value of PLR, MLR, and NWR levels on prognosis was analyzed. (4) Patients were divided into high-level group and low-level group according to PLR, MLR, and NWR values; survival curves of patients with different PLR, MLR, and NWR values were analyzed; and survival rates of patients with different PLR, MLR, and NWR values were compared.

RETRACTED

### 2.6. Statistical Methods

All data in this study were input into EXCEL table by two people without communication and were analyzed and processed by statistical software SPSS24.0. Measurement data were expressed as mean ± SD ($\bar{\text{x}}\pm s$). The data consistent with normal distribution and homogeneity of variance were statistically analyzed by *t*-test, and one-way ANOVA was used for data comparison between multiple groups. Counting data were described by *n* and %, chi-square test was used for comparison between groups, and rank sum test was used for comparison of ranked data. ROC curve was used to analyze the evaluation value of PLR, MLR, and NWR levels on the clinical efficacy of neoadjuvant chemotherapy in patients with locally advanced gastric cancer. GraphPad Prism5 was used for image and survival curve analysis; log-rank *χ*^2^ test was used to analyze the survival rate between the two groups. All were two-sided tests, and *P* < 0.05 was considered statistically significant.

## 3. Results

### 3.1. Comparison of PLR, MLR, and NWR Values between the Effective Group and the Ineffective Group

The effective rate of neoadjuvant chemotherapy in patients with locally advanced gastric cancer was 62.60% (82/131), and the PLR, MLR, and NWR values in the effective group were lower than those in the ineffective group (*P* < 0.05), as shown in Figure 1.

(Note: Comparison of PLR, MLR, and NWR values between the two groups, ^∗^ indicated *P* < 0.05)

### 3.2. The Evaluation Value of PLR, MLR, and NWR Values for Clinical Efficacy

The AUC of combined PLR, MLR, and NWR in evaluating the efficacy of neoadjuvant chemotherapy was greater than that of PLR and NWR alone (*P* < 0.05), as shown in Table 1 and Figure 2.

### 3.3. Comparison of PLR, MLR, and NWR Values in Patients with Different Clinical Stages

The PLR value of patients with stage IIIa, IIIb, and IIIc was higher than that of patients with stage II, the MLR value of patients with stage IIIb and IIIc was greater than that of patients with stage II and IIIa, and the NMR value of patients with stage IIIc was greater than that of patients with stage II, IIIa, and IIIb (*P* < 0.05), see Figure 3.

### 3.4. Correlation Analysis of PLR, MLR, and NWR Values and Clinical Stage

PLR, MLR, and NWR values were positively correlated with clinical stage (*P* < 0.05), as shown in Figure 4.

### 3.5. Comparison of PLR, MLR, and NWR Values between the Survival Group and Death Group

The PLR, MLR, and NWR values of the survival group were lower than those of the death group (*P* < 0.05), as shown in Figure 5.

(Note: Comparison of PLR, MLR, and NWR values between the two groups, ^∗^ indicated *P* < 0.05)

RETRACTED

### 3.6. Predictive Value of PLR, MLR, and NWR Values for Prognosis

The AUC of combined PLR, MLR, and NWR in predicting the prognosis of patients was greater than that of MLR and NWR alone (*P* < 0.05), as shown in Table 2 and Figure 6.

### 3.7. Survival Curve Analysis of Patients with Different PLR, MLR, and NWR Values

The survival rate of patients with PLR ≥ 162.11 (36.21%, 21/58) was lower than that of patients with PLR < 162.11 (80.82%, 59/73) (log-rank *χ*^2^ = 23.431, *P* < 0.05), and the survival rate of patients with MLR ≥ 0.31 (42.86%, 24/56) was lower than that of patients with MLR < 0.31 (74.67%, 56/75) (log-rank *χ*^2^ = 12.523, *P* < 0.05), and the survival rate of patients with NWR ≥ 0.62 (45.00%, 27/60) was lower than NWR < 0.62 patients (74.65%, 53/71) (log-rank *χ*^2^ = 9.613, *P* < 0.05), see Figure 7.

## 4. Discussion

Locally advanced gastric cancer refers to gastric cancer that only invades the liver, pancreas, and other surrounding organs or has local lymph node metastasis, localized to the periphery of the tumor, but without distant lymph node metastasis. In the past, surgical resection was generally abandoned and only gastric jejunostomy was used for conservative treatment, but the therapeutic effect was poor [11]. Relevant studies have pointed out that the 3-year survival rate of palliative resection for localized advanced gastric cancer is low and the prognosis of patients is poor [12]. Therefore, how to convert inoperable or potentially resectable gastric cancer into operable resection through appropriate preoperative treatment is the most urgent problem in the treatment of gastric cancer. Neoadjuvant chemotherapy can not only shrink the primary tumor and lymph nodes but also eliminate potential metastatic lesions, thereby reducing the stage, prolonging the survival period of patients, and improving the quality of life of patients [13]. Studies have found that preoperative neoadjuvant chemotherapy and postoperative combined organ resection can significantly improve the survival rate of patients with tumor invading surrounding organs and distant metastasis [14, 15]. In this study, neoadjuvant chemotherapy was applied in the clinical treatment of locally advanced gastric cancer, and it was found that the effective rate of neoadjuvant chemotherapy was 62.60%, which was not much different from relevant studies [16], but much higher than palliative treatment efficacy. Therefore, it may be feasible to apply this therapy to locally advanced gastric cancer. In this study, for patients with stable efficacy or disease progression confirmed by CT reexamination after neoadjuvant chemotherapy treatment, considering that tumor cells may be resistant to neoadjuvant chemotherapy drugs, chemotherapy regimen should be changed in the follow-up treatment to improve clinical benefit rate and prognosis of patients. Therefore, for patients receiving neoadjuvant chemotherapy, CT examination should be conducted regularly before and during treatment, and treatment plan should be adjusted timely according to the patient's situation.

RETRACTED

In recent years, studies have found that inflammatory response and tissue carcinogenesis share similar molecular targets and signaling pathways [17]. Inflammation is involved in the construction of tumor microenvironment by changing tumor tissue homeostasis. In recent years, more and more scholars have found that abnormal levels of inflammatory cells and immunomodulatory molecules exist in various tumor microenvironments, which can affect tumor progression and metastasis [18]. Inflammation can lead to abnormal immune function of the body, resulting in a decrease in the number of lymphocytes. Relevant reports point out that the production of a large number of inhibitory immune cells, neutrophils, etc. can promote inflammatory responses, mediate tumor cell proliferation and angiogenesis, and lead to further tumor infiltration or metastasis [19, 20]. Neutrophils can promote tumor growth and metastasis by upregulating the expression of related proteases and cytokines. In addition, neutrophils can promote the growth of tumor cells by reshaping extracellular matrix and releasing reactive oxygen species. Effective chemotherapy can eliminate the influence of tumor on the body to a certain extent. At present, changes in tumor size are often used to evaluate clinical treatment effect, and changes in tumor microenvironment are also closely related to tumor growth and reproduction. Therefore, this study suggests that the tumor environment before treatment may also be related to the therapeutic effect of neoadjuvant chemotherapy. This study found that PLR, MLR, and NWR values in the effective group were lower than those in the ineffective group, indicating that the inflammatory state of the body was related to the clinical treatment effect, which is mainly related to the aggravated inflammatory response, and can promote further tumor metastasis, and then affect the clinical treatment [21, 22]. Further analysis in this study found that the AUC of combined PLR, MLR, and NWR in evaluating the efficacy of neoadjuvant chemotherapy was greater than that of PLR and NWR alone, and the AUC value was greater than 0.8, indicating that the combined detection has evaluation value for the efficacy of neoadjuvant chemotherapy, so it may be applied in the treatment evaluation of locally advanced gastric cancer.

RETRACTED

Tumor-associated inflammatory cells can release a series of inflammatory mediators, cytokines, and enzymes, resulting in changes in vascular permeability, which can aggravate local inflammatory responses and can cause oxidative damage and changes in the tumor microenvironment by releasing inflammatory mediators, thus promoting the proliferation and metastasis of tumor cells [23]. Relevant studies have pointed out that changes in local inflammatory state of the body may be related to tumor progression [24]. The results of this study showed that PLR, MLR, and NWR values were positively correlated with clinical stage, indicating that the increase of PLR, MLR, and NWR values may be related to tumor progression. It is currently believed that neutrophils and platelets in the tumor microenvironment are involved in the occurrence and development of tumors and play an important role in tumor-related inflammation and immunity. Relevant reports pointed out that the increase of peripheral blood neutrophils is related to the hematopoietic cytokines produced by tumors [25]. Platelets can promote the growth and metastasis of cancer cells by promoting angiogenesis and producing adhesion molecules, reduce the damage of immune attack and mechanical injury to cancer cells, assist cancer cells to escape from immune, and then promote tumor progression or metastasis.

With tumor progression and metastasis, neutrophil and platelet counts in patients increase, and the body's inflammatory response and antitumor immunity are abnormal, which promotes tumor cell infiltration and metastasis. Relevant reports indicate that changing the preoperative inflammatory state and immune state can effectively improve the long-term prognosis of patients with malignant tumor [26]. Cancer cells can induce platelet aggregation, and tissue factor secreted by cancer cells can also promote platelet production and activation. Neutrophils can promote angiogenesis and tissue infiltration by secreting vascular endothelial factor and matrix protease, thereby promoting tumor occurrence, invasion, and metastasis, and the increase of neutrophil count can directly affect the body's NWR value. NLR can reflect the body's tumor inflammation and immune status. Relevant studies have pointed out that high level of NLR is conducive to promoting tumor cell proliferation and metastasis, resulting in poor prognosis [27, 28]. In this study, the PLR, MLR, and NWR values in the survival group were lower than those in the death group, and the survival rates of patients with PLR ≥ 162.11, MLR ≥ 0.31, and NWR ≥ 0.62 were lower than those with PLR < 162.11, MLR < 0.31, and NWR < 0.62, respectively, suggesting that the prognosis of patients was related to the changes of PLR, MLR, and NWR values. The reason is that when NLR and PLR increase, the body's effective defense is weakened, and the barrier against malignant tumor cells is destroyed, thus affecting the prognosis of patients [29]. In addition, the results of this study showed that the AUC of combined PLR, MLR, and NWR values in evaluating the prognosis of patients was greater than that of MLR and NWR alone, indicating that combined detection has predictive value for the prognosis of patients. The patients with different PLR, MLR, and NWR values were followed up to the end point of the study, and the survival curve analysis was performed. The results showed that patients with PLR ≥ 162.11 or MLR ≥ 0.31 or NWR ≥ 0.62 had a lower survival rate (follow-up 3 years). The results provide some guidance for predicting the prognosis of patients with locally advanced gastric cancer by neoadjuvant chemotherapy using PLR, MLR, and NWR. However, this study still needs a larger sample size and more in-depth research to support this conclusion.

RETRACTED

In conclusion, PLR, MLR, and NWR values are correlated with clinical stage, and combined detection has evaluation value for the clinical efficacy of neoadjuvant chemotherapy and prediction value for the prognosis of locally advanced gastric cancer patients. However, there are still shortcomings in this study. This study is a single-center retrospective study, and the statistical results may be biased. Therefore, multicenter analysis is needed to further explore the relationship between PLR, MLR, and NWR values and this disease.

## Figures and Tables

**Figure 1:** Comparison of PLR, MLR, and NWR values between the effective group and the ineffective group.

**Figure 2:** ROC curve analysis of PLR, MLR, and NWR values for evaluating clinical efficacy.

**Figure 3:** Comparison of PLR, MLR, and NWR values in patients with different clinical stages.

**Figure 4:** Correlation analysis between PLR, MLR, and NWR values and clinical stages.

**Figure 5:** Comparison of PLR, MLR and NWR values between the survival group and death group.

**Figure 6:** ROC curve analysis of PLR, MLR, and NWR values in predicting prognosis of patients.

**Figure 7:** Survival curve analysis of patients with different PLR, MLR, and NWR values.

**Table 1:** The evaluation value of PLR, MLR, and NWR values for clinical efficacy.

Indicator	Cutoff value	AUC	SE	95% CI
PLR	159.85	0.759^∗^	0.044	0.673~0.846
MLR	0.31	0.809	0.040	0.730~0.888
NWR	0.64	0.737^∗^	0.043	0.652~0.822
Combination		0.889	0.030	0.830~0.947

Note: ^∗^ indicated *P* < 0.05 when compared with combination.

**Table 2:** Predictive value of PLR, MLR, and NWR values for prognosis.

Indicator	Cutoff value	AUC	SE	95% CI
PLR	162.11	0.747	0.044	0.660~0.834
MLR	0.31	0.727^∗^	0.044	0.640~0.814
NWR	0.62	0.675^∗^	0.048	0.581~0.769
Combination		0.805	0.038	0.731~0.880

Note: ^∗^ indicated *P* < 0.05 when compared with combination.

RETRACTED

## Data Availability

The labeled datasets used to support the findings of this study are available from the corresponding author upon request.

## References

[1] Wang C. (2021). The effect of total parenteral nutrition support on the immune function of patients after radical gastrectomy for gastric cancer: a review of immunotherapy of cancer: immunosuppression and tumor growth (2nd edition). *Chinese Experimental Formulary Journal*.

[2] Wang Y., Zhang J., Guo S., Li X. K., Fan Q. X. (2020). Indications of neoadjuvant chemotherapy for locally advanced gastric cancer patients based on pre-treatment clinicalpathological and laboratory parameters. *Journal of Cancer*.

[3] Kyh A., Mts A., Jjb A. (2019). Use of neoadjuvant chemotherapy in the treatment of locally advanced rectal cancer - Science Direct. *Journal of Surgical Research*.

[4] (2013). National Health and Family Planning Commission of the People's Republic of China. Guidelines for standardized diagnosis and treatment of gastric cancer (trial). *Journal of Chronic Diseases*.

[5] Lv Q., Xia Q., Li A., Wang Z. (2021). The potential role of IL1RAP on tumor microenvironment-related inflammatory factors in stomach adenocarcinoma. *Technology in Cancer Research & Treatment*.

[6] Zhu Z. Y., Wang Y. M., Li F. K. (2020). Prognostic evaluation of platelet-to-lymphocyte ratio and neutrophil-to-lymphocyte ratio in patients with TNM stage I to III gastric cancer. *Zhonghua Digestion Journal*.

[7] Feng F., Sun L., Zheng G. (2017). Low lymphocyte-to-white blood cell ratio and high monocyte-to-white blood cell ratio predict poor prognosis in gastric cancer. *Oncotarget*.

[8] Wang F. H., Zhang X. T., Li Y. F. (2021). The Chinese Society of Clinical Oncology (CSCO): clinical guidelines for the diagnosis and treatment of gastric cancer, 2021. *Cancer Communications*.

[9] (2020). National Comprehensive Cancer Network. Gastric cancer, version 3.2020, NCCN clinical practice guidelines in oncology. *Journal of the National Comprehensive Cancer Network Jnccn*.

[10] Yang X. N., Wu Y. L. (2004). Evaluation criteria for treatment of solid tumors-RECIST. *Evidence-Based Medicine*.

[11] Choi Y. W., Ahn M. S., Jeong G. S. (2019). The role of surgical resection before palliative chemotherapy in advanced gastric cancer. *Scientific Reports*.

[12] Zheng Y., Zhang X. J., Shi B. Q., Zhang W., Wang L., Chao L. M. (2020). Clinical observation of quality of life and anxiety in elderly patients with advanced gastric cancer before and after different palliative interventional treatments. *Journal of Interventional Radiology*.

RETRACTED

[13] Peng L. Q., Yang W., Zhang Z. D. (2018). Propensity score matching prognostic analysis of neoadjuvant chemotherapy for locally advanced gastric cancer. *Chinese Journal of Gastrointestinal Surgery*.

[14] Chen T., Ning J., Campisi A. (2022). Neoadjuvant PD-1 inhibitors and chemotherapy for locally advanced NSCLC: a retrospective study. *Ann Thorac*.

[15] Shen Z., Tian L., Wang X. (2018). Treatment of pancreatic head cancer with obstructive jaundice by endoscopy ultrasonography-guided gastrojejunostomy. *Medicine*.

[16] Ding P. A., Zhang Z. D., Tan B. B. (2021). Prediction of the efficacy and prognosis of neoadjuvant chemotherapy for advanced gastric cancer by systemic inflammatory response index-prognostic nutritional index score role. *Chinese Journal of Experimental Surgery*.

[17] Wang J. L., Liu F. X., Zhao Y. Y., Wei M. J., He M. (2019). Analysis of miRNAs with potential biomarker properties and their target gene biological functions and signaling pathways in prostate cancer tissue. *Shandong Medicine*.

[18] Wu D. H., Zhang S. G., Liu L. X. (2018). The mechanism of action of neutrophil extracellular traps in tumor formation. *Journal of University of Science and Technology of China*.

[19] Dymicka-Piekarska V., Koper-Lenkiewicz O. M., Zińczuk J., Kratz E., Kamińska J. (2021). Inflammatory cell-associated tumors. Not only macrophages (TAMs), fibroblasts (TAFs) and neutrophils (TANs) can infiltrate the tumor microenvironment. The unique role of tumor associated platelets (TAPs). *Cancer Immunology, Immunotherapy*.

[20] Jia X. Y., Guo Z. C., Sun Y., Gong Z. C. (2021). Study on the ability of CXC chemokine ligand 2 to promote the invasion ability of oral squamous cell carcinoma in tumor microenvironment by recruiting tumor-associated neutrophils. *Journal of Practical Stomatology*.

[21] Chen Q., Wang J., Zhang Q., Zhang J., Bai X. (2019). Tumour cell-derived debris and IgG synergistically promote metastasis of pancreatic cancer by inducing inflammation via tumour-associated macrophages. *British Journal of Cancer*.

[22] Yang L. Y., Luo Q., Lu L. (2020). Increased neutrophil extracellular traps promote metastasis potential of hepatocellular carcinoma via provoking tumorous inflammatory response. *Journal of Hematology & Oncology*.

[23] Li S., Zhou J., Zhao P., He Q., Luo H. C. (2021). The relationship between preoperative neutrophil-to-lymphocyte-to-platelet-to-lymphocyte ratio and C-reactive protein to albumin ratio and postoperative lymph node metastasis in patients with cN0 gastric cancer. *China Clinical Oncology*.

RETRACTED

[24] Zhu J., Lian L., Qin H. (2019). Prognostic evaluation of patients with resectable lung cancer using systemic inflammatory response parameters. *Oncology Letters*.

[25] Xia T. S., Liu B. T., Wang F. J. (2017). The value of preoperative peripheral blood neutrophil to lymphocyte ratio and platelet to lymphocyte ratio in evaluating lymph node metastasis in patients with gastric cancer. *Zhonghua Digestive Journal*.

[26] Johnson S. C., Chakraborty S., Drosou A. (2020). Inflammatory state of lymphatic vessels and miRNA profiles associated with relapse in ovarian cancer patients. *PLoS One*.

[27] Wang S., Liang C. C., Zhou J., Shi H. Q., Yang C., Wang J. Z. (2019). The value of neutral-lymphocyte ratio and prognostic nutritional index in the prognosis evaluation of patients with radical bladder cancer. *Journal of Anhui Medical University*.

[28] Jiang D. P., Xu H. P., Fang H. J., Zhao G. H. (2020). Analysis of related factors affecting the prognosis of patients after radical gastrectomy. *China Modern Medical Journal*.

[29] Hu G., Li W., Shao G. Y., Zhang X. (2018). The predictive value of preoperative platelet to lymphocyte ratio in patients with gastric stromal tumor. *Cancer Prevention and Treatment Research*.

